The article "Identification of Cuproptosis-Related Genes in Nonalcoholic Fatty Liver Disease" was published in 2023. Journal: Oxid Med Cell Longev.

# Identification of Cuproptosis-Related Genes in Nonalcoholic Fatty Liver Disease

**DOI:** 10.1155/2023/9245667

**Published:** 2023-02-21

**Authors:** Chutian Wu, Xiongxiu Liu, Lixian Zhong, Yun Zhou, Linjing Long, Tingzhuang Yi, Sisi Chen, Yuting Li, Yanfang Chen, Lianli Shen, Qiuting Zeng, Shaohui Tang

**Affiliations:** ^1^Department of Gastroenterology, The First Affiliated Hospital, Jinan University, Guangzhou, Guangdong 510630, China; ^2^Department of Gastroenterology, The First Affiliated Hospital, Gannan Medical University, Ganzhou 341000, China; ^3^Department of Gastroenterology, The Fifth Affiliated Hospital, Guangzhou Medical University, Guangzhou, Guangdong 510700, China; ^4^Department of Oncology, Affiliated Hospital of YouJiang Medical University For Nationalities, Baise, Guangxi 533000, China

## Abstract

Nonalcoholic fatty liver disease (NAFLD) is the most prevalent hepatic pathology worldwide. However, the precise molecular mechanisms for NAFLD are still not sufficiently explained. Recently, a new mode of cell death (cuproptosis) is found. However, the relationship between NAFLD and cuproptosis remains unclear. We analyzed three public datasets (GSE89632, GSE130970, and GSE135251) to identify cuproptosis-related genes stably expressed in NAFLD. Then, we performed a series of bioinformatics analyses to explore the relationship between NAFLD and cuproptosis-related genes. Finally, 6 high-fat diet- (HFD-) induced NAFLD C57BL/6J mouse models were established to carry out transcriptome analysis. The results of gene set variation analysis (GSVA) revealed that the cuproptosis pathway was abnormally activated to a certain degree (*p* = 0.035 in GSE89632, *p* = 0.016 in GSE130970, *p* = 0.22 in GSE135251), and the principal component analysis (PCA) of the cuproptosis-related genes showed that the NAFLD group separated from the control group, with the first two principal components accounting for 58.63%-74.88% of the variation. Among three datasets, two cuproptosis-related genes (*DLD* and *PDHB*, *p* < 0.01 or 0.001) were stably upregulated in NAFLD. Additionally, both *DLD* (AUC = 0.786–0.856) and *PDHB* (AUC = 0.771–0.836) had favorable diagnostic properties, and the multivariate logistics regression model further improved the diagnostic properties (AUC = 0.839–0.889). NADH, flavin adenine dinucleotide, and glycine targeted *DLD*, and pyruvic acid and NADH targeted *PDHB* in the DrugBank database. The *DLD* and *PDHB* were also associated with clinical pathology, especially with steatosis (*DLD*, *p* = 0.0013–0.025; *PDHB*, *p* = 0.002–0.0026) and NAFLD activity score (*DLD*, *p* = 0.004–0.02; *PDHB*, *p* = 0.003–0.031). What is more, *DLD* and *PDHB* were correlated with stromal score (*DLD*, *R* = 0.38, *p* < 0.001; *PDHB*, *R* = 0.31, *p* < 0.001) and immune score (*DLD*, *R* = 0.26, *p* < 0.001; *PDHB*, *R* = 0.27, *p* < 0.001) in NAFLD. Furthermore, *Dld* and *Pdhb* were also significantly upregulated in the NAFLD mouse model. In conclusion, cuproptosis pathways, especially *DLD* and *PDHB*, could be potential candidate genes for NAFLD diagnostic and therapeutic options.

The article "Identification of Cuproptosis-Related Genes in Nonalcoholic Fatty Liver Disease" was published in 2023. Journal: Oxid Med Cell Longev.

## 1. Introduction

Nonalcoholic fatty liver disease (NAFLD), as a metabolic disease, is the most prevalent hepatic pathology worldwide with a prevalence of approximately 25% [1]. It ranges from simple steatosis (SS) to advanced stage of nonalcoholic steatohepatitis (NASH), the latter rapid progression toward liver cirrhosis, and hepatocellular carcinoma (HCC) [2, 3]. Currently, sensitive biomarkers for the diagnosis of NAFLD are still lacking, and liver biopsies, as an invasive method, are still considered the gold standard for diagnosis and prognosis [4]. Although numerous studies have attempted to study the pathogenesis and progression of NAFLD, there are still no effective drugs for NAFLD other than lifestyle changes [5]. Moreover, the development of NAFLD is a complex process and is still not sufficiently explained [6]. Consequently, it is crucial to explore the mechanisms involved in the pathogenesis of NAFLD to identify new potential targets for diagnosis and therapy.

Recently, Tsvetkov et al. [7] have shown a new mode of cell death, copper-dependent cell death, which is called “cuproptosis.” It can be simply summarized that copper directly binds to lipoylated components of the tricarboxylic acid (TCA) cycle and subsequent Fe-S cluster protein loss causes proteotoxic stress that triggers cell death [8]. The expression changes of ten genes (known as cuproptosis-related genes) involve in cuproptosis, among which seven genes (ferredoxin 1 (*FDX1*), lipoyl synthase (*LIAS*), lipolytransferas 1 (*LIPT1*), dihydrolipoamide dehydrogenase (*DLD*), dihydrolipoamide S-acetyltransferase (*DLAT*), pyruvate dehydrogenase E1 subunit alpha 1 (*PDHA1*), and pyruvate dehydrogenase E1 subunit beta (*PDHB*)) were upregulated, and three genes (metal-regulatory transcription factor 1 (*MTF1*), glutaminase (*GLS*), and cyclin-dependent kinase inhibitor 2A (*CDKN2A*)) were downregulated [7].

There has been recognition that copper metabolism disorder can lead to a variety of chronic liver diseases, such as Wilson disease (WD), NAFLD, and liver cirrhosis [9]. Zhang et al. indicated that serum copper levels were positively correlated with body mass index (BMI), leptin, and insulin resistance, which are all risk factors for NAFLD [2]. Dev et al. found a dramatic increase in hepatic copper levels, resulting in obesity and hepatic steatosis in the hepatocyte-specific knockout of *Atp7b* WD mouse model [10].

The article "Identification of Cuproptosis-Related Genes in Nonalcoholic Fatty Liver Disease" was published in 2023. Journal: Oxid Med Cell Longev.

In this research, we seek to comprehensively investigate the molecular alterations and clinical relevance of the cuproptosis-related genes in NAFLD. This study highlights the importance of cuproptosis-related genes in NAFLD and lays a foundation for future studies of cuproptosis in NAFLD.

## 2. Materials and Methods

### 2.1. Data Retrieving and Processing from GEO

Data from Gene Expression Omnibus (GEO, http://www.ncbi.nlm.nih.gov/geo) fulfilled the inclusion criteria below: ① publication date from 2010 to 2022; ② containing NAFLD and normal tissue samples; ③ providing detailed clinicopathological information. The exclusion criteria were as follows: ① duplicated research; ② patients who underwent bariatric surgery or with severe diseases; ③ data that could not be analyzed; ④ animal or cell experiments. Subsequently, the gene expression profiles of GSE89632 [11], GSE130970 [12], and GSE135251 [13] were downloaded from GEO. Eventually, 24 control patients, 19 SS patients, and 19 NASH patients in GSE89632, 6 control patients and 72 NAFLD patients in GSE130970, 10 control patients, and 216 NAFLD patients were included in this study (Table 1). Since the datasets were from a public database, patient consent and ethics committee approval were not required. Then, the gene array data (GSE89632) was converted into the quantile normalized values, and the read count data (GSE130970 and GSE135251) was standardized by the transcripts per million (TPM). The overall research design is shown in Figure 1.

### 2.2. Gene Set Variation Analysis (GSVA) and Single-Sample Gene Set Enrichment Analysis (ssGSEA)

GSVA, a pathway enrichment method that estimated variation of pathway activity, was performed to evaluate the role of the cuproptosis pathway in NAFLD using R package “GSVA” [14]. In addition, the stromal score, immune score, and immune cells' marker enrichment were ssGSEA and they were calculated by “estimate” (http://bioinformatics.mdanderson.org/estimate/), and “GSVA” R packages. The immune gene sets were downloaded from Charoentong et al. [15]. Then, the spearman correlation analysis between *DLD*/*PDHB* expression and immune cells was performed. The results were visualized using the “ggplot2” R package.

### 2.3. Correlation Analysis of Cuproptosis-Related Genes, Protein-Protein Interaction (PPI) Network Construction, and the Prediction of Potential Drugs

The “ggcorrplot” R package was used to recognize the correlation between cuproptosis-related genes by the Spearman correlation analysis. The STRING database (https://string-db.org/) was utilized to construct a PPI network with an interaction score > 0.4. The prediction of potential drugs was performed in the DrugBank database (https://go.drugbank.com).

The article "Identification of Cuproptosis-Related Genes in Nonalcoholic Fatty Liver Disease" was published in 2023. Journal: Oxid Med Cell Longev.

### 2.4. Gene Ontology (GO) and Kyoto Encyclopedia of Genes and Genomes (KEGG) Analyses

To explore the potential pathways of *DLD* and *PDHB*, the GO and KEGG analyses were performed using “clusterProfiler” [16] and “org.Hs.eg.db” R package. The median of the risk model scores of *DLD* and *PDHB* was selected as the cut-off value.

### 2.5. Animal Model and Experiment Design

A total of 6 male C57BL/6J mice (weight, 23.47 ± 1.18 g; age, 6 weeks) were purchased from the medical laboratory animal center of Guangdong (Guangzhou, China). All the mice were acclimatized under a temperature of 24 ± 2°C, a relative humidity of 55 ± 10%, and a 12 h light/dark cycle for 10 days before the commencement of the animal experiment. All animal experiments were approved by the experimental animal ethics committee of Jinan University and were performed in accordance with the Guidelines for Care and Use of Laboratory Animals of Jinan University (IACUC-20190916-09).

After acclimation, the 6 mice were randomly divided into the normal control group (NC, *n* = 3) and the NAFLD group (*n* = 3). The NC group mice were fed with standard mouse diet, and the NAFLD group mice were induced by a high-fat diet (HFD) (containing 34% fat, 2% cholesterol, 26% carbohydrate, 26% protein, and 12% basic feed (*w*/*w*)) for 8 weeks before sacrificing.

### 2.6. Histological Analysis

At the end of the study, the mice were sacrificed to measure liver mass and liver mass index by using the following formula: live mass index = liver mass/body mass × 100%. Afterward, the liver samples were immersed in 10% formalin neutral buffer solution for 48 h, then processed routinely, embedded in paraffin, sectioned to 5 *μ*m thickness and stained with hematoxylin and eosin (H&E). Lipid accumulation in liver was analyzed by Oil red O (ORO) staining (Sigma). Slides were observed with a light microscope (Leica DMi 8).

### 2.7. Transcriptome Analysis of Mice Liver Tissues

The quality and integrity of total RNA were supervised on Agilent Technologies 2100 Bioanalyzer (Agilent Technologies, Waldbronn, Germany). The RNA sequencing library was generated from 250 ng total RNA using Ribo-off rRNA Depletion Kit (Vazyme BioTech, Nanjing, China) for rRNA depletion followed by VAHTSⓇ Universal V6 RNA-seq Library Prep Kit RNA Library Prep Kit for Illumina (Vazyme BioTech, Nanjing, China) according to the manufacturer's protocols. The libraries were sequenced on Illumina NovaSeq 6000 (Illumina, California, USA). Sequences were aligned to the mm10 mouse reference genome using STAR Aligner. Then, reads aligning to genes were counted using htseq-count, and analysis of differentially expressed genes (DEGs) was performed using the “limma” R package [17] and later visualized by volcano plot using “ggplot2” R package (https://ggplot2.tidyverse.org/). The threshold for the DEGs was set as *p* value < 0.05 and |log_2_ fold change (FC)| ≥ 0.5. The raw data was stored in the ArrayExpress database (accession: E-MTAB-11980, https://www.ebi.ac.uk/arrayexpress/).

The article "Identification of Cuproptosis-Related Genes in Nonalcoholic Fatty Liver Disease" was published in 2023. Journal: Oxid Med Cell Longev.

### 2.8. Statistical Analysis

Statistical analysis was performed using R software (Version 4.1.3, http://www.r-project.org). Statistical comparisons between two groups of continuous data were performed using the *t*-test or Mann–Whitney *U*-test according to the test condition and the Kruskal-Wallis test for multiple comparisons among the groups. Principal component analysis (PCA) was applied to display the overall differences of cuproptosis-related genes and visualized by the “ggplot2” R package. Venn diagram was performed using the “ggvenn” R package. The multivariate logistics regression risk model was constructed in *DLD* and *PDHB*. A receiver-operating characteristic (ROC) curve was conducted to assess the diagnostic value of the genes and the model by “pROC” R package and visualized by the “ggplot2” R package. A difference with *p* < 0.05 was considered significant.

## 3. Results

### 3.1. Cuproptosis Pathway Plays a Role in NALFD

To determine whether the cuproptosis pathway played a role in NAFLD, GSVA and PCA were performed. The results showed that the enrichment score of the cuproptosis pathways in GSE89632 and GSE130970 was significantly increased (*p* < 0.05) in the NAFLD group compared with the control group, but not in GSE135251 (*p* = 0.22, Figures 2(a)–2(c)). Next, the principal component analysis (PCA) of the cuproptosis-related genes showed that the NAFLD group separated from the control group, with the first two principal components accounting for 58.63%-74.88% of the variation (Figures 2(d)–2(f)). These results suggest that the cuproptosis pathway is activated to some degree in NAFLD.

### 3.2. Differential Expression of Cuproptosis-Related Genes

Subsequently, the expression levels of the cuproptosis-related genes were explored in the three datasets, respectively. The cuproptosis-related genes were changed to varying degrees in the three datasets, in which *DLD* (*p* < 0.001 in GSE89632, *p* = 0.004 in GSE130970, *p* < 0.001 in GSE135251) and *PDHB* (*p* = 0.001 in GSE89632, *p* = 0.007 in GSE130970, *p* = 0.001 in GSE135251) were stably and significantly upregulated in the three datasets (Figures 3(a)–3(d)). The outcomes illustrate that *DLD* and *PDHB* play a part in the pathogenesis and progression of NAFLD.

The article "Identification of Cuproptosis-Related Genes in Nonalcoholic Fatty Liver Disease" was published in 2023. Journal: Oxid Med Cell Longev.

### 3.3. Correlation Analysis of Cuproptosis-Related Genes and PPI Network Construction

The Spearman correlation analysis showed that there were potential interactions between the cuproptosis-related genes (Figures 3(e) and 3(f)). Moreover, *DLD* and *PDHB* both had strong correlations in the three datasets (*R* = 0.51, *p* < 0.0001 in GSE89632; *R* = 0.53, *p* < 0.0001 in GSE130970; *R* = 0.77, *p* < 0.0001 in GSE135251). Afterward, the PPI analysis further suggested the potential interactions among them. *DLD* and *PDHB* had more PPI edges than other genes, suggesting that *DLD* and *PDHB* were hub genes (Figure 3(h)).

### 3.4. *DLD* and *PDHB* Are Associated with Clinical Characteristics of NAFLD and the Prediction of Potential Drugs

Next, we further explored the relationship between *DLD*/*PDHB* and clinical characteristics, respectively. First, the diagnostic values of *DLD* and *PDHB* were evaluated through ROC analysis. By observing the area under the curve (AUC), both *DLD* and *PDHB* had favorable diagnostic properties (AUC = 0.786/0.771 in GSE89632, AUC = 0.856/0.836 in GSE130970, and AUC = 0.837/0.802 in GSE135251) (Figures 4(a)–4(c)). Then, GSE130970 was used for the training set and GSE135251 for the testing set. The multivariate logistics regression model further improved the diagnostic properties (AUC = 0.889 in GSE130970 and AUC = 0.839 in GSE135251), and the risk model was summarized using the following equation: Response = −1.63 + 0.24^∗^log_2_(DLD [TPM] + 1) + 0.20^∗^ log_2_(PDHB [TPM] + 1) (Figures 4(b) and 4(c)). These results indicate that *DLD* and *PDHB* may be potential biomarkers in the diagnosis of NAFLD.

After that, the association between *DLD*/*PDHB* and clinical pathology was analyzed separately. In GSE89632, *DLD* was significantly positively associated with steatosis (*p* = 0.0013), ballooning (*p* = 0.028), lobular inflammation (*p* = 0.048), and NAS (*p* = 0.02) (Figure 4(d)); *PDHB* was significantly positively relative to steatosis (*p* = 0.002), ballooning (*p* = 0.027), NAS (*p* = 0.031), and fibrosis (*p* = 0.034) (Figure 4(e)). In GSE130970, *DLD* was significantly positively associated with steatosis (*p* = 0.025), lobular inflammation (*p* = 0.007), and fibrosis (*p* = 0.0064) (Figure 4(f)); *PDHB* was only significantly positively relative to steatosis (*p* = 0.0026) (Figure 4(g)). In GSE135251, both *DLD* (*p* = 0.004) and *PDHB* (*p* = 0.003) were positively associated with NAS, but not fibrosis (Figure 4(h)). We then predicted the potential drugs for *DLD* and *PDHB* in the DrugBank database and showed that nicotinamide adenine dinucleotide (NADH), flavin adenine dinucleotide (FAD), glycine targeted *DLD*, and pyruvic acid and NADH targeted *PDHB* (Figure 4(i)). All in all, *DLD* and *PDHB* are associated with the clinical pathology of NAFLD.

The article "Identification of Cuproptosis-Related Genes in Nonalcoholic Fatty Liver Disease" was published in 2023. Journal: Oxid Med Cell Longev.

### 3.5. *DLD* and *PDHB* Are Associated with Metabolic Pathways and Copper Toxicity

Subsequently, GO and KEGG analyses were implemented for pathway analysis by comparing the low- and high-risk scores of *DLD* and *PDHB* in GSE130970. The GO results showed that the high-risk score of *DLD* and *PDHB* was associated with the acetyl-CoA metabolic process and fatty acid metabolic process, and detoxification of copper ion pathway was enriched in the low-risk score group (Figure 5(a)). Besides, the KEGG results illustrated that the high-risk score of *DLD* and *PDHB* was associated with fatty acid metabolism, glycolysis/gluconeogenesis, and pyruvate metabolism (Figure 5(b)). These results indicate that high-expressed *DLD* and *PDHB* appear to increase copper toxicity and are related to the acetyl-CoA metabolic process and pyruvate metabolism, both important substrate sources for the TCA cycle.

### 3.6. *DLD* and *PDHB* Are Positively Correlated with Stromal Score and Immune Score

Considering that GSE135251 had the largest sample size, we chose it to explore the relationship between the *DLD*/*PDHB* and the immune microenvironment. *DLD* was positively correlated with stromal score (*R* = 0.38, *p* = 7.18*e*^−09^, Figure 6(a)) and immune score (*R* = 0.26, *p* = 9.15*e*^−05^, Figure 6(b)). Meanwhile, *DLD* was positively associated with multiple immune cells, especially with gamma delta T cell, CD4+ T cell, and immature dendritic cell (*R* > 0.3, *p* < 0.05, Figure 6(c)). On the other hand, *PDHB* was also positively correlated with stromal score (*R* = 0.31, *p* = 4.89*e*^−06^, Figure 6(d)) and immune score (*R* = 0.27, *p* = 7.34*e*^−05^, Figure 6(e)). *PDHB* was also positively associated with multiple immune cells, especially with memory CD4 T cell, gamma delta T cell, and immature dendritic cell (*R* > 0.3, *p* < 0.05, Figure 6(f)). These results indicate that *DLD* and *PDHB* have an impact on the immune microenvironment.

### 3.7. Further Validation of *DLD* and *PDHB* in the NAFLD Mouse Model

Mice fed HFD develop hepatic steatosis, mimicking the NAFLD of humans [18]. We conducted an animal experiment, and after HFD was fed to NAFLD mouse group for 8 weeks, a significant increase in the body mass, liver mass, and liver mass index was observed in the NAFLD group compared with the NC group (Table 2). Besides, the results of liver pathology showed that liver sections from the NALFD group had hepatocyte swelling, ballooning degeneration, and different sizes of lipid droplets (Figures 7(a) and 7(b)). Oil Red O staining revealed the accumulation of neutral lipids in NAFLD (Figures 7(c) and 7(d)). These results demonstrate that the NAFLD mouse model was successfully established.

The article "Identification of Cuproptosis-Related Genes in Nonalcoholic Fatty Liver Disease" was published in 2023. Journal: Oxid Med Cell Longev.

Subsequently, transcriptome analysis of mice liver tissues indicated that *Dld* and *Pdhb* were also significantly upregulated in the NAFLD group compared with the NC group (Figure 7(e)).

## 4. Discussion

In this study, we first explored the relationship between 10 cuproptosis-related genes and NAFLD. Then, *DLD* and *PDHB* were stably upregulated in NAFLD among the three datasets. Besides, the *DLD* and *PDHB* were also associated with the clinical characteristics (especially steatosis and NAS) and the immune microenvironment in NAFLD. NADH, FAD, and glycine targeted *DLD*, and pyruvic acid and NADH targeted *PDHB*. In addition, the high-expressed *DLD* and *PDHB* appeared to increase copper toxicity and had impacts on the TCA cycle by affecting the acetyl-CoA and pyruvate, further suggesting that the cuproptosis might affect the development of NAFLD. Furthermore, the NAFLD mouse model was established to determine the expression signature of *Dld* and *Pdhb*. These outcomes suggest that *DLD* and *PDHB* promoted hepatic steatosis and trigger liver inflammation through the cuproptosis.

Copper, a cofactor for various enzymes, is an essential micronutrient required for normal cell function, and the cuproptosis is related to various cancer progressions, such as HCC [19, 20]. Recent studies have determined that serum and liver copper are related to NAFLD, but the specific mechanism is still unclear [21]. Mitochondrial respiration is required for cuproptosis, but upregulation of mitochondrial activity often occurs in an early NAFLD stage, and the expression levels of cuproptosis-related genes (*DLD* and *PDHB*) are increased in our study, which suggests that cuproptosis may contribute to the progression of NAFL to NASH [7, 22]. However, the mitochondrial function gradually decreases during the progression of NAFLD, suggesting that the effect of cuproptosis is progressively attenuated and may lead to HCC eventually [22]. In addition, it is reported that suppression of *DLD* expression inhibits melanoma growth and tumor proliferation by increasing intracellular reactive oxygen species (ROS) production and thereby inducing autophagy cell death [23]. *PDHB* catalyzes the conversion of pyruvate to acetyl-CoA, acting as a central node that links glucose metabolism, lipid metabolism, and the TCA [24]. The dysfunction of *PDHB* can lead to metabolism alteration which is one of the hallmarks of cancer cells [25, 26]. Recent studies show that glycine and hepatic NAD^+^ decrease in NAFLD individuals, and their supplementation can ameliorate NAFLD, but their mechanisms have not been completely elucidated, and our study may provide new insight for them [27–29]. Besides, the altered pyruvate metabolism, particularly enhanced lactate production, plays an essential role in the NAFLD progression, but further studies are needed to determine whether pyruvic acid supplementation improves NAFLD [30]. FAD, a redox-active coenzyme, is involved in various metabolic pathways, including the beta-oxidation of fatty acid and TCA, and its role in NAFLD is still unknown [31]. Moreover, *DLD* and *PDHB* are positively correlated with gamma delta T cell and CD4+ T cell which often accumulate in the liver and subsequent stimulate inflammatory processes in NAFLD [32, 33]. Hence, the cuproptosis, especially *DLD* and *PDHB*, may also play a vital role in NAFLD.

The article "Identification of Cuproptosis-Related Genes in Nonalcoholic Fatty Liver Disease" was published in 2023. Journal: Oxid Med Cell Longev.

The present study had several advantages. Firstly, this was the first study to explore the relationship between NAFLD and cuproptosis-related genes. Secondly, we comprehensively analyzed multiple datasets and screened out stably upregulated cuproptosis-related genes (*DLD* and *PDHB*), which were later verified in the NAFLD mouse model, whereas our study also had some limitations. First of all, we did not carry out an in-depth study of cuproptosis on NAFLD. For another, the NAFLD mouse model rather than human tissue was used in this study, which might have influenced the results. But HFD-induced NAFLD mouse model can mimic the NAFLD of humans most accurately [18].

In conclusion, our study presented a systematic analysis of molecular alterations and interactive genes of cuproptosis in NAFLD. Finally, we screened out two cuproptosis-related genes (*DLD* and *PDHB*) that were correlated with NAFLD prognosis. Although further research is still needed, we provide useful and novel information to explore the potential candidate genes for NAFLD diagnostic and therapeutic options.

## Figures and Tables

**Figure 1:** The overall research design. The data were downloaded from the GEO database. Then, GSVA and PCA were performed to identify the activation of the cuproptosis pathway in NAFLD. The differential expression analysis (DEA) and Venn diagram showed that *DLD* and *PDHB* were stably upregulated in three datasets. Subsequently, correlation analysis and PPI were conducted to explore their relationship. Clinical pathology analysis and risk model construction were carried out. Next, the immune microenvironment and potential drugs for *DLD* and *PDHB* were explored. Finally, the NAFLD mouse model was used to further verify the expression of *DLD* and *PDHB*.

The article "Identification of Cuproptosis-Related Genes in Nonalcoholic Fatty Liver Disease" was published in 2023. Journal: Oxid Med Cell Longev.

**Figure 2:** Gene set variation analysis (GSVA) of cuproptosis pathways in GSE89632 (a), GSE130970 (b), and GSE135251 (c); principal component analysis (PCA) of cuproptosis-related genes in GSE89632 (d), GSE130970 (e), and GSE135251 (f). SS: simple steatosis; NAFLD: nonalcoholic fatty liver disease; NASH: nonalcoholic steatohepatitis.

**Figure 3:** The expression levels of 10 cuproptosis-related genes in GSE89632 (a), GSE130970 (b), and GSE135251 (c); (d) the Venn diagram shown the overlap of the three datasets, and *DLD* and *PDHB* were selected. Correlations among the expression of cuproptosis-related genes in GSE89632 (e), GSE130970 (f), and GSE135251 (g); (h) protein-protein interaction (PPI) analysis further confirmed the correlations between cuproptosis-related genes. ^∗^*p* < 0.05; ^∗∗^*p* < 0.01; ^∗∗∗^*p* < 0.001; ^∗∗∗∗^*p* < 0.0001; ns: not significance; Corr: correlation *R*; SS: simple steatosis; NAFLD: nonalcoholic fatty liver disease; NASH: nonalcoholic steatohepatitis.

**Figure 4:** The receiver-operating characteristic (ROC) curve examined the diagnostic value of *DLD*/*PDHB* in GSE89632 (a), GSE130970 (b), and GSE135251 (c); the relationship between *DLD* (d)/*PDHB* (e) and clinicopathology in GSE89632; the relationship between *DLD* (f)/*PDHB* (g) and clinicopathology in GSE130970; (h) the relationship between *DLD*/*PDHB* and clinicopathology in GSE130970; (i) potential therapeutic agents of *DLD* and *PDHB*. AUC: area under the curve; NAS: NAFLD activity score; NADH: nicotinamide adenine dinucleotide; FAD: flavin adenine dinucleotide.

**Figure 5:** Enrichment plots of GO (a) and KEGG (b) showing the related signaling pathways of the risk model of *DLD* and *PDHB.*

**Figure 6:** *DLD* was positively correlation with stromal score (a) and immune score (b); (c) correlation analysis between *DLD* and the immune cells. *PDHB* was positively correlation with stromal score (d) and immune score (e); (f) correlation analysis between *PDHB* and the immune cells.

**Figure 7:** The hematoxylin and eosin (H&E) staining of NC mouse ((a) ×400) and NAFLD mouse ((b) ×400); the Oil red O (ORO) staining of NC mouse ((c) ×400) and NAFLD mouse ((d) ×400); (e) the volcano plot shown the differential expressed genes in the NAFLD mouse group compare with the NC group.

**Table 1:** Clinical characteristics of the datasets.

Items	Control	SS	NASH
*GSE89632*			
*n*	24	20	19
Male, *n* (%)	11 (45.8%)	14 (70.0%)	9 (47.4%)
Age, median (IQR)	38 (26.8-46.3)	45.5 (36.5-51.3)	44 (35.5-51.5)
NAS			
<3	24	17	0
3-4	0	3	9
>4	0	0	10
Steatosis			
0	24	0	0
1	0	10	6
2	0	7	7
3	0	3	6
Ballooning			
0	24	20	0
1	0	0	13
2	0	0	6
Lobular inflammation			
0	24	20	0
1	0	0	11
2	0	0	6
3	0	0	2
Fibrosis			
0	18	17	4
1-2	6	3	7
3-4	0	0	8
*GSE130970*	Control	NAFLD	
*n*	6	72	
Male, *n* (%)	2 (33.3%)	28 (38.9%)	
Age, median (IQR)	61 (34.5-63.5)	52 (42.5-57.5)	
NAS			
<3	6	11	
3-4	0	35	
>4	0	26	
Steatosis			
0	6	2	
1	0	29	
2	0	27	
3	0	14	
Ballooning			
0	6	14	
1	0	28	
2	0	30	
Lobular inflammation			
0	6	5	
1	0	55	
2	0	12	
3	0	0	
Fibrosis			
0	6	19	
1-2	6	37	
3-4	0	16	
*GSE135251*	Control	NAFLD	
*n*	10	206	
NAS			
<3	10	32	
3-4	0	64	
>4	0	110	
Fibrosis			
0	8	38	
1-2	2	100	
3-4	0	68	

IQR: interquartile range; SS: simple steatosis; NASH: nonalcoholic steatohepatitis; NAS: NAFLD activity score.

The article "Identification of Cuproptosis-Related Genes in Nonalcoholic Fatty Liver Disease" was published in 2023. Journal: Oxid Med Cell Longev.

**Table 2:** The conditions of NAFLD mouse.

Items	NC	NAFLD	*p* value
Day 1 weight (g)	22.71 ± 0.77	24.22 ± 1.10	0.125
Week 8 weight (g)	27.17 ± 0.60	36.53 ± 1.85	0.001
Liver mass (g)	0.92 ± 0.06	1.74 ± 0.18	0.002
Liver mass index (%)	3.40 ± 0.19	4.75 ± 0.36	0.005

The data are shown as mean ± standard deviation. NC: normal control group; NAFLD: nonalcoholic fatty liver disease group.

## Data Availability

The data can be found in ArrayExpress and GEO databases, accession numbers: E-MTAB-11980, GSE89632, GSE130970, and GSE135251. The coding can be found on GitHub (https://github.com/biomedt/oxidative/tree/main).
